# A Mathematical Model of COVID-19 Pandemic: A Case Study of Bangkok, Thailand

**DOI:** 10.1155/2021/6664483

**Published:** 2021-03-30

**Authors:** Pakwan Riyapan, Sherif Eneye Shuaib, Arthit Intarasit

**Affiliations:** Department of Mathematics and Computer Science, Faculty of Science and Technology, Prince of Songkla University, Pattani Campus, Pattani 94000, Thailand

## Abstract

In this study, we propose a new mathematical model and analyze it to understand the transmission dynamics of the COVID-19 pandemic in Bangkok, Thailand. It is divided into seven compartmental classes, namely, susceptible (*S*), exposed (*E*), symptomatically infected (*I*_*s*_), asymptomatically infected (*I*_*a*_), quarantined (*Q*), recovered (*R*), and death (*D*), respectively. The next-generation matrix approach was used to compute the basic reproduction number denoted as *R*_cvd19_ of the proposed model. The results show that the disease-free equilibrium is globally asymptotically stable if *R*_cvd19_ < 1. On the other hand, the global asymptotic stability of the endemic equilibrium occurs if *R*_cvd19_ > 1. The mathematical analysis of the model is supported using numerical simulations. Moreover, the model's analysis and numerical results prove that the consistent use of face masks would go on a long way in reducing the COVID-19 pandemic.

## 1. Introduction

The world continues to battle with the coronavirus disease 2019 (COVID-19) caused by the novel coronavirus, SARS-CoV-2, which is regarded as a highly virulent virus that targets the human respiratory system. The pandemic started in late December 2019 with patients admitted to hospitals with an initial diagnosis of pneumonia. The admitted patients' sickness was linked to the seafood and wet animal market in Wuhan, Hubei Province, China [1]. On January 2, 2020, a total number of 41 admitted hospital patients were confirmed to be infected with COVID-19 [2]. On January 22, 2020, 571 COVID-19 cases were reported in 25 different provinces in China [1, 2]. On January 30, 2020, China had about 7734 confirmed COVID-19 cases, while 90 cases were reported in about 13 countries [1, 3], including Canada, India, Germany, France, the United States, India, and the United Arab Emirates. As of October 31, 2020, a total of 4,667,780 COVID-19 cases (Africa: 1,776,595 cases, Asia: 13,461,293 cases, America: 20,546,580 cases, Europe: 9,840,736 cases, Oceania: 41,880 cases, and others: 696 cases) have been reported worldwide including 1,189,499 deaths (Africa: 42,688 deaths, Asia: 239,675 deaths, America: 640,513 deaths, Europe: 265,565 deaths, Oceania: 1,051 deaths, and others: 7 deaths) [4].

COVID-19 is transmitted from human to human via direct contact with contaminated surfaces and through respiratory droplets' inhalation from infected individuals [5]. Presently, there is no vaccine or antiviral treatment approved for the prevention or management of COVID-19 [6]. To effectively reduce the spread of COVID-19, governments have been implementing various control measures such as imposing strict, mandatory lockdowns and encouraging (and in some cases strictly enforcing) other measures such as individuals maintaining a minimum distance between themselves (social distancing), avoiding crowded events, imposing a maximum number of individuals in any gathering (religious and social), and the use of face masks in public [7]. To further help mitigate the spread of COVID-19, contact tracing of suspected infected cases has been stepped up in several countries and detected cases (asymptomatic and symptomatic) are quickly placed in isolation for prompt treatment [7].

In Thailand, the virus was first confirmed to exist on January 13, 2020 [8], while the first reported local transmission was confirmed on January 31, 2020 [9]. The number of cases remained low throughout February, but it surged in mid-March. The rise in the number of cases was traced to several transmission clusters, the largest of which occurred with a Muay Thai fight at the military-run Lumpinee Boxing Stadium on March 6, 2020 [10]. Confirmed cases rose to over a hundred per day over the following week, and public venues and businesses were ordered to close in Bangkok and several other provinces [11]. Bangkok businesses' abrupt closure prompted tens of thousands of workers to travel to their hometowns [12]. The Prime Minister of Thailand, Prayut Chan-o-cha, declared a state of emergency, effective on March 26, 2020 [13], and a curfew went into effect on April 3, 2020 [14]. All commercial international flights were suspended from April 4, and lockdown measures were implemented in varying degrees throughout the country. The rate of new cases gradually dropped throughout April, and by mid-May, locally transmitted infection rates had fallen to near-zero, and easing of restrictions was gradually implemented [15, 16].

Even though there had been no new domestic cases since mid-May, on August 21, Thailand extended its emergency degree until September 30 to prevent incoming aliens from overseas in many routes. In September, a prison inmate who had not been abroad was Thailand's first locally transmitted case in 100 days. Later in the month, Akbar Ismatullaev, a footballer, was infected with the virus after completing the 14-day state quarantine since he arrived nearly a month earlier. In October, foreign tourists entered Thailand for the first time in seven months [17]. A French tourist on Ko Samui in Surat Thani contracted the disease after passing the 14-day state quarantine. She developed a fever 17 days after arriving in the country. In October, foreign tourists entered Thailand for the first time in seven months under the Special Tourist Visa program [18].

Mathematical modeling is a valuable tool to control disease spread effectively. Several useful mathematical models have been formulated in the last few decades to study infectious diseases and develop helpful strategies for the efficient elimination of infection [19–25]. The compartmental models and real cases are more effective in providing valuable information about a particular disease outbreak. Several mathematical models have already been formulated in various countries to analyze the complex transmission pattern of the COVID-19 pandemic, using ordinary differential equations [26–28], delay differential equations [29], stochastic differential equations [30], and fractional order Caputo derivative [31–36].

Thailand has begun opening its borders to foreigners and with the growing cases in the USA and Europe, there is a concern that COVID-19 cases in Thailand may rise soon. Hence, this study is aimed at (i) formulating a mathematical model to understand the dynamics of the COVID-19 pandemic in Bangkok, Thailand, (ii) examining the impact of the control measures currently employed in Thailand, and (iii) determining if these measures will be effective in preventing COVID-19 cases in Thailand. The remainder of this article is structured as follows. The proposed model is presented in Mathematical Model Formulation and Description. The mathematical analysis of the model is presented in Analysis of the Model. The results obtained from numerical simulations of the model are provided in Numerical Simulation. Finally, the conclusion drawn from this study is given in Conclusion.

## 2. Mathematical Model Formulation and Description

The mathematical model of COVID-19 transmission formulated in this study was motivated by the study of [26]. The model proposed in [26] was constructed from the SEIR model and is comprised of six compartments with the infected compartment divided into three categories. However, in the present study, the model will be divided into seven compartments. The total human population to be considered is denoted as *N*(*t*), and at any time, it comprises of the susceptible (*S*), exposed (*E*), symptomatically infected (*I*_*s*_), asymptomatically infected (*I*_*a*_), quarantined (*Q*), recovered (*R*), and death (*D*) compartments, respectively. The susceptible compartment comprises individuals living in the country or who have recently returned before the border's closure. The individuals exposed to COVID-19 and show signs of symptoms are moved to the symptomatic infectious compartment. In contrast, individuals who show no sign of symptoms are moved to the asymptomatic infectious compartment. There is a reduction in the risk of infection for the individuals in the susceptible compartment since they practice preventive measures such as social distancing, wearing a mask, and refraining from mass gatherings or meetings. Individuals move to the recovery compartment through recovery from both the quarantined and infected compartments, respectively. The parameters *β*_*s*_ and *β*_*a*_, respectively, represent the effective contact rate (contacts capable of leading to COVID-19 transmission) for individuals in the symptomatically infectious and asymptomatically infectious compartments. The proportion of individuals who wear face masks correctly within a community is denoted as 0 < *ψ* ≤ 1 while 0 < *ξ* ≤ 1 represent the expected decrease in the risk of infection due to the face mask's use. The progression rate of exposed individuals is denoted as *φ*. A proportion 0 < *θ* ≤ 1 of exposed individuals showed no clinical symptoms of COVID-19 (and move to the compartment *I*_*a*_) at the end of the incubation period. The remaining proportion 1 − *θ* shows clinical symptoms and moves to the *I*_*s*_ compartment. The parameters*λ*_*s*_, *λ*_*a*_, and *λ*_*q*_ represent the recovery rate for individuals in *I*_*s*_,*I*_*a*_, and *Q* compartments, respectively. Similarly, *α*_*s*_ and *α*_*a*_ are the isolation rate of individuals. Finally, the parameters *δ*_*s*_ and *δ*_*q*_ represent the COVID-19-induced mortality rate for individuals in the asymptomatic infectious and quarantined compartments, respectively. In this study, the effect of social distancing and community lockdown measures will be measured based on the overall reduction in the community contact rate parameter's baseline values.

The flowchart of the formulated model using all the above assumptions is given in Figure 1. Additionally, all variables with their meaning and the parameters with their description are provided in Tables 1 and 2, respectively.

From the above assumptions and variables, we formulate the model with nonnegative initial conditions:

(1) $$\begin{array}{c} \frac{dS}{dt}=\rho -\beta_{s}\left(1-\psi \xi \right){SI}_{s}-\beta_{a}\left(1-\psi \xi \right){SI}_{a}-\mu S,\\ \frac{dE}{dt}=\beta_{s}\left(1-\psi \xi \right){SI}_{s}+\beta_{a}\left(1-\psi \xi \right){SI}_{a}-\left(\varphi +\mu \right)E,\\ \frac{{dI}_{s}}{dt}=\left(1-\theta \right)\varphi E-\left(\alpha_{s}+\delta_{s}+\lambda_{s}+\mu \right)I_{s},\\ \frac{{dI}_{a}}{dt}=\theta \varphi E-\left(\alpha_{a}+\lambda_{a}+\mu \right)I_{a},\\ \frac{dQ}{dt}=\alpha_{s}I_{s}+\alpha_{a}I_{a}-\left(\lambda_{q}+\delta_{q}+\mu \right)Q,\\ \frac{dR}{dt}=\lambda_{s}I_{s}+\lambda_{a}I_{a}+\lambda_{q}Q-\mu R,\\ \frac{dD}{dt}=\delta_{s}I_{s}+\delta_{q}Q. \end{array}$$

Since the total population is *N*(*t*) = *dS*/*dt* + *dE*/*dt* + *dI*_*s*_/*dt* + *dI*_*a*_/*dt* + *dQ*/*dt* + *dR*/*dt* + *dD*/*dt*, then

(2) $$\begin{array}{c} N\left(t\right)=\rho -\mu N. \end{array}$$

From (2), *N*(*t*) would approach a carrying capacity *ρ*/*μ*. Model (1) describes the human population, and thus, the model variables can be shown to be nonnegative for all time *t* ≥ 0 and that all solutions of the model (1) will remain positive for all time *t* ≥ 0. Therefore, model (1) is mathematically well-posed, and its dynamics can be considered in the region below:

(3) $$\begin{array}{c} \Omega_{\text{Cvd}19}=\left\{\left(S,E,I_{s},I_{a},Q,R,D\right)\in R_{+}^{7}:S+E+I_{s}+I_{a}+Q+R+D\leq \frac{\rho }{\mu }\right\}. \end{array}$$

## 3. Analysis of Model (1)

In this section, the dynamical properties of model (1) are qualitatively studied.

### 3.1. Positivity and Boundedness of Solutions

Since model (1) illustrates the human population, it is important that model (1) is epidemiologically meaningful and all states of variables are nonnegative for all time *t* > 0. Using Theorem 1, the positivity of solutions of model (1) is first discussed below.

**Theorem 1 .**

If *S*(0) > 0, *E*(0) > 0, *I*_*s*_(0) > 0, *I*_*a*_(0) > 0, *Q*(0) > 0, *R*(0) > (0) and *D*(0) > 0, then the solutions (*S*(*t*) > 0, *E*(*t*) > 0, *I*_*s*_(*t*) > 0, *I*_*a*_(*t*) > 0, *Q*(*t*) > 0, *R*(*t*) > 0, *D*(*t*) > 0) of the model are positive for all time *t* > 0.

**Proof**

From the first equation of the model, we have that

(4) $$\begin{array}{c} \frac{dS}{dt}=\rho -\beta_{s}\left(1-\psi \xi \right){SI}_{s}-\beta_{a}\left(1-\psi \xi \right){SI}_{a}-\mu S\geq -\beta_{s}\left(1-\psi \xi \right){SI}_{s}-\beta_{a}\left(1-\psi \xi \right){SI}_{a}-\mu S. \end{array}$$

By using the technique of variable separation, *dS*/*dt* can be reduced to

(5) $$\begin{array}{c} \frac{dS}{dt}\geq -\beta_{s}\left(1-\psi \xi \right){SI}_{s}-\beta_{a}\left(1-\psi \xi \right){SI}_{a}-\mu S. \end{array}$$

Then, the above equation is integrated to yield the solution below

(6) $$\begin{array}{c} S\left(t\right)\geq S_{0}{\text{e}}^{-\int_{0}^{t}\left(\beta_{s}\left(1-\psi \xi \right)I_{s}+\beta_{a}\left(1-\psi \xi \right)I_{a}+\mu \right)dS}>0. \end{array}$$

Since the initial value *S*_0_ and the exponential functions in Equation (6) are always positive. Hence, *S*(*t*) is positive. Using the same ideas to check other equations of model (1), this shows that *E*(*t*) > 0, *I*_*s*_(*t*) > 0, *I*_*a*_(*t*) > 0, *Q*(*t*) > 0, *R*(*t*) > 0, *D*(*t*) > 0. Next, using Theorem 2, we prove the boundedness of the nonnegative solutions characterized by Theorem 1.

**Theorem 2 .**

All positive solutions described in Theorem 1 are bounded.

**Proof**

The addition of all equations in Equation (1) yields

(7) $$\begin{array}{c} \frac{dN}{dt}=\frac{d}{dt}\left(S+E+I_{s}+I_{a}+Q+R+D\right)=\rho -\mu N, \end{array}$$

which can be rewritten as

(8) $$\begin{array}{c} N\left(t\right)=\frac{\rho }{\mu }-\left[\frac{\rho -\rho N_{0}}{\rho }\right]e^{-\mu t}. \end{array}$$

From Equation (8), *N*(*t*) approaches *ρ*/*μ* as *t* → ∞. Hence, the positive solutions of model (1) are bounded.

### 3.2. The Equilibrium Points of Model

The equilibrium points of model (1) are obtained by zeroing the right-hand side of all equations in model (1), resulting in

(9) $$\begin{array}{c} \rho -\beta_{s}\left(1-\psi \xi \right){SI}_{s}-\beta_{a}\left(1-\psi \xi \right){SI}_{a}-\mu S=0,\\ \beta_{s}\left(1-\psi \xi \right){SI}_{s}+\beta_{a}\left(1-\psi \xi \right){SI}_{a}-\left(\varphi +\mu \right)E=0,\\ \left(1-\theta \right)\varphi E-\left(\alpha_{s}+\delta_{s}+\lambda_{s}+\mu \right)I_{s}=0,\\ \theta \varphi E-\left(\alpha_{a}+\lambda_{a}+\mu \right)I_{a}=0,\\ \alpha_{s}I_{s}+\alpha_{a}I_{a}-\left(\lambda_{q}+\delta_{q}+\mu \right)Q=0,\\ \lambda_{s}I_{s}+\lambda_{a}I_{a}+\lambda_{q}Q-\mu R=0,\\ \delta_{s}I_{s}+\delta_{q}Q=0. \end{array}$$

The simplification of Equation (9) can yield many solutions. However, in this study, we consider two solutions: the disease-free equilibrium point (DFEP) and the endemic equilibrium point (EEP). The DFEP in this study is denoted as *χ*_dfep_^∗^ = (*S*_dfep_^∗^, *E*_dfep_^∗^, *I*_*s*_^∗^_dfep_, *I*_*a*_^∗^_dfep_, *Q*_dfep_^∗^, *R*_dfep_^∗^, *D*_dfep_^∗^), where

(10) $$\begin{array}{c} S_{\text{dfep}}^{*}=\frac{\rho }{\mu },\\ E_{\text{dfep}}^{*}=0,\\ {I_{s}^{*}}_{\text{dfep}}=0,\\ {I_{a}^{*}}_{\text{dfep}}=0,\\ Q_{\text{dfep}}^{*}=0,\\ R_{\text{dfep}}^{*}=0,\\ D_{\text{dfep}}^{*}=0. \end{array}$$

Furthermore, the EEP is denoted by *χ*_eep_^∗^ = (*S*_eep_^∗^, *E*_eep_^∗^, *I*_*s*_^∗^_eep_, *I*_*a*_^∗^_eep_, *Q*_eep_^∗^, *R*_eep_^∗^, *D*_eep_^∗^), where

(11) $$\begin{array}{c} S_{\text{eep}}^{*}=\frac{\rho }{\beta_{s}\left(1-\psi \xi \right)I_{s}+\beta_{a}\left(1-\psi \xi \right)I_{a}+\mu },\\ E_{\text{eep}}^{*}=\frac{\beta_{s}\left(1-\psi \xi \right)I_{s}+\beta_{a}\left(1-\psi \xi \right)I_{a}}{\varphi +\mu },\\ {I_{s}^{*}}_{\text{eep}}=\frac{\left(1-\theta \right)\varphi E}{\alpha_{s}+\delta_{s}+\lambda_{s}+\mu },\\ {I_{a}^{*}}_{\text{eep}}=\frac{\theta \varphi E}{\alpha_{a}+\lambda_{a}+\mu },\\ Q_{\text{eep}}^{*}=\frac{\alpha_{s}I_{s}+\alpha_{a}I_{a}}{\lambda_{q}+\delta_{q}+\mu },\\ R_{\text{eep}}^{*}=\frac{\lambda_{s}I_{s}+\lambda_{a}I_{a}+\lambda_{q}Q}{\mu Q},\\ D_{\text{eep}}^{*}=0. \end{array}$$

### 3.3. The Basic Reproduction Number of Model (1)

To compute the model's basic reproduction number (BRN), the next-generation matrix approach is employed. In this study, we denote the BRN of model (1) as *R*_cvd19_, which is defined as the number of secondary cases of COVID-19 infection arising from one individual infected with the COVID-19 disease. By using the notation in the study of [37], the vectors *ℱ* (denotes new infection) and *𝒱* (transfer of individuals between compartments) are given as follows:

(12) $$\begin{array}{c} F=\left(\begin{array}{c} \beta_{s}{SI}_{s}\left(1-\psi \xi \right)+\beta_{a}{SI}_{a}\left(1-\psi \xi \right)\\ 0\\ 0 \end{array}\right),\\ V=\left(\begin{array}{c} \left(\varphi +\mu \right)E\\ -\left(1-\theta \right)\varphi E+\left(\alpha_{s}+\delta_{s}+\lambda_{s}+\mu \right)I_{s}\\ -\theta \varphi E+\left(\alpha_{a}+\lambda_{a}+\mu \right)I_{a} \end{array}\right). \end{array}$$

From vectors *ℱ* and *𝒱*, the Jacobian *F* and *𝒱* are computed below:

(13) $$\begin{array}{c} F=\left(\begin{array}{ccc} 0 & \beta_{s}S\left(1-\psi \xi \right) & \beta_{a}S\left(1-\psi \xi \right)\\ 0 & 0 & 0\\ 0 & 0 & 0 \end{array}\right),\\ V=\left(\begin{array}{ccc} \left(\varphi +\mu \right) & 0 & 0\\ -\left(1-\theta \right)\varphi & \left(\alpha_{s}+\delta_{s}+\lambda_{s}+\mu \right) & 0\\ -\theta \varphi & 0 & \alpha_{a}+\lambda_{b}+\mu \end{array}\right). \end{array}$$

The Jacobian matrices *F* and *V* evaluated at *χ*_eep_^∗^ yield:

(14) $$\begin{array}{c} F=\left(\begin{array}{ccc} 0 & \beta_{s}S_{\text{dfep}}^{*}\left(1-\psi \xi \right) & \beta_{a}S_{\text{dfep}}^{*}\left(1-\psi \xi \right)\\ 0 & 0 & 0\\ 0 & 0 & 0 \end{array}\right),\\ V=\left(\begin{array}{ccc} \left(\varphi +\mu \right) & 0 & 0\\ -\left(1-\theta \right)\varphi & \left(\alpha_{s}+\delta_{s}+\lambda_{s}+\mu \right) & 0\\ -\theta \varphi & 0 & \left(\alpha_{a}+\lambda_{a}+\mu \right) \end{array}\right). \end{array}$$

Hence, computing the Jacobian matrices *F* and *V*, the BRN of the model is

(15) $$\begin{array}{c} R_{\text{cvd}19}=\rho \left({FV}^{-1}\right)=\frac{\varphi S_{\text{dfep}}^{*}}{\varphi +\mu }\left[\frac{\beta_{s}\left(1-\psi \xi \right)\left(1-\theta \right)}{\alpha_{s}+\delta_{s}+\lambda_{s}+\mu }+\frac{+{\theta \beta }_{a}\left(1-\psi \xi \right)}{\left(\alpha_{a}+\lambda_{a}+\mu \right)}\right], \end{array}$$

where *S*_dfep_^∗^ is denoted in Equation (10).

From Equation (15), the BRN of model (1) can be further simplified to Equation (16):

(16) $$\begin{array}{c} R_{\text{cvd}19}=\frac{\beta_{s}\varphi S_{\text{dfep}}^{*}\left(1-\psi \xi \right)\left(1-\theta \right)}{\varphi +\mu \left(\alpha_{s}+\delta_{s}+\lambda_{s}+\mu \right)}+\frac{{\theta \beta }_{a}\varphi S_{\text{dfep}}^{*}\left(1-\psi \xi \right)}{\varphi +\mu \left(\alpha_{a}+\lambda_{a}+\mu \right)}. \end{array}$$

Equation (16) comprises two reproduction numbers. The first BRN is (*β*_*s*_*φS*_dfep_^∗^(1 − *ψξ*)(1 − *θ*))/(*φ* + *μ*(*α*_*s*_ + *δ*_*s*_ + *λ*_*s*_ + *μ*)), and it defines the number of new COVID-19 cases generated from symptomatically infectious human in compartment *I*_*s*_. The second BRN is (*θβ*_*a*_*φS*_dfep_^∗^(1 − *ψξ*))/(*φ* + *μ*(*α*_*a*_ + *λ*_*a*_ + *μ*)), and it defines the number of new COVID-19 cases generated from asymptomatically infectious humans in compartment *I*_*a*_. Hence, mathematically, the BRN can be simplified to be

(17) $$\begin{array}{c} R_{\text{cvd}19}={RI}_{s}+{RI}_{a}. \end{array}$$

## 4. Global Stability Analysis

### 4.1. Global Stability Analysis of DFEP

To prove the global stability of the disease-free equilibrium, the Lyapunov function below is constructed:

(18) $$\begin{array}{c} L=B_{1}E+B_{2}I_{s}+B_{3}I_{a}, \end{array}$$

where

(19) $$\begin{array}{c} B_{1}=\left(\alpha_{a}+\lambda_{a}+\mu \right)\left(\alpha_{s}+\delta_{s}+\lambda_{s}+\mu \right),\\ B_{2}=\left(\alpha_{a}+\lambda_{a}+\mu \right)\beta_{s}\left(1-\psi \xi \right)S,\\ B_{3}=\left(\alpha_{s}+\delta_{s}+\lambda_{s}+\mu \right)\beta_{a}\left(1-\psi \xi \right)S. \end{array}$$

From Equation (18), the derivative is given below as

(20) $$\begin{array}{c} \frac{\partial L}{\partial t}=B_{1}\frac{dE}{dt}+B_{2}\frac{{dI}_{s}}{dt}+B_{3}\frac{{dI}_{a}}{dt}=B_{1}\left[\beta_{s}\left(1-\psi \xi \right){SI}_{s}+\beta_{a}\left(1-\psi \xi \right){SI}_{a}-\left(\varphi +\mu \right)E\right]+B_{2}\left[\left(1-\theta \right)\varphi E-\left(\alpha_{s}+\delta_{s}+\lambda_{s}+\mu \right)I_{s}\right]+B_{3}\left[\theta \varphi E-\left(\alpha_{a}+\lambda_{a}+\mu \right)I_{a}\right]. \end{array}$$

The expansion of Equation (20) yields

(21) $$\begin{array}{c} \frac{\partial L}{\partial t}=\left(\alpha_{a}+\lambda_{a}+\mu \right)\left(\alpha_{s}+\delta_{s}+\lambda_{s}+\mu \right)\left[\beta_{s}\left(1-\psi \xi \right){SI}_{s}+\beta_{a}\left(1-\psi \xi \right){SI}_{a}-\left(\varphi +\mu \right)E\right]+\left(\alpha_{a}+\lambda_{a}+\mu \right)\beta_{s}S\left(1-\psi \xi \right)\left[\left(1-\theta \right)\varphi E-\left(\alpha_{s}+\delta_{s}+\lambda_{s}+\mu \right)I_{s}\right]+\left(\alpha_{s}+\delta_{s}+\lambda_{s}+\mu \right)\beta_{a}S\left(1-\psi \xi \right)\left[\theta \varphi E-\left(\alpha_{a}+\lambda_{a}+\mu \right)I_{a}\right]. \end{array}$$

Then, Equation (21) becomes

(22) $$\begin{array}{c} \frac{\partial L}{\partial t}=\left(\alpha_{a}+\lambda_{a}+\mu \right)\left(\alpha_{s}+\delta_{s}+\lambda_{s}+\mu \right)\left[\beta_{s}\left(1-\psi \xi \right){SI}_{s}\right]-\left(\alpha_{a}+\lambda_{a}+\mu \right)\beta_{s}S\left(1-\psi \xi \right)\left(\alpha_{s}+\delta_{s}+\lambda_{s}+\mu \right)+\left(\alpha_{a}+\lambda_{a}+\mu \right)\left(\alpha_{s}+\delta_{s}+\lambda_{s}+\mu \right)\left[\beta_{a}\left(1-\psi \xi \right){SI}_{a}\right]-\left(\alpha_{s}+\delta_{s}+\lambda_{s}+\mu \right)\beta_{a}S\left(1-\psi \xi \right)\left(\alpha_{a}+\lambda_{a}+\mu \right)+\left(\alpha_{a}+\lambda_{a}+\mu \right)\beta_{s}S\left(1-\psi \xi \right)\left(1-\theta \right)\varphi E+\left(\alpha_{s}+\delta_{s}+\lambda_{s}+\mu \right)\beta_{a}\left(1-\psi \xi \right)\theta \varphi E-\left(\alpha_{a}+\lambda_{a}+\mu \right)\left(\alpha_{s}+\delta_{s}+\lambda_{s}+\mu \right)\left(\varphi +\mu \right)E. \end{array}$$

Equation (22) can be simplified to

(23) $$\begin{array}{c} \frac{\partial L}{\partial t}=\left(\alpha_{a}+\lambda_{a}+\mu \right)\left(\alpha_{s}+\delta_{s}+\lambda_{s}+\mu \right)\left[\beta_{s}\left(1-\psi \xi \right){SI}_{s}\right]-\left(\alpha_{a}+\lambda_{a}+\mu \right)\beta_{s}S\left(1-\psi \xi \right)\left(\alpha_{s}+\delta_{s}+\lambda_{s}+\mu \right)+\left(\alpha_{a}+\lambda_{a}+\mu \right)\left(\alpha_{s}+\delta_{s}+\lambda_{s}+\mu \right)\left[\beta_{a}\left(1-\psi \xi \right){SI}_{a}\right]-\left(\alpha_{s}+\delta_{s}+\lambda_{s}+\mu \right)\beta_{a}S\left(1-\psi \xi \right)\left(\alpha_{a}+\lambda_{a}+\mu \right)+\left(\alpha_{a}+\lambda_{a}+\mu \right)\left(\alpha_{s}+\delta_{s}+\lambda_{s}+\mu \right)\left(\varphi +\mu \right)\left[\frac{\beta_{s}S\left(1-\psi \xi \right)\left(1-\theta \right)\varphi }{\left(\varphi +\mu \right)\left(\alpha_{s}+\delta_{s}+\lambda_{s}+\mu \right)}+\frac{\beta_{a}\left(1-\psi \xi \right)\theta \varphi }{\left(\varphi +\mu \right)\left(\alpha_{a}+\lambda_{a}+\mu \right)}-1\right]E,\\ \frac{\partial L}{\partial t}\leq \left(\alpha_{a}+\lambda_{a}+\mu \right)\left(\alpha_{s}+\delta_{s}+\lambda_{s}+\mu \right)\left(\varphi +\mu \right)\left[\frac{\beta_{s}S\left(1-\psi \xi \right)\left(1-\theta \right)\varphi }{\left(\varphi +\mu \right)\left(\alpha_{s}+\delta_{s}+\lambda_{s}+\mu \right)}+\frac{\beta_{a}\left(1-\psi \xi \right)\theta \varphi }{\left(\varphi +\mu \right)\left(\alpha_{a}+\lambda_{a}+\mu \right)}-1\right]E\leq \left(\alpha_{a}+\lambda_{a}+\mu \right)\left(\alpha_{s}+\delta_{s}+\lambda_{s}+\mu \right)\left(\varphi +\mu \right)\left[R_{\text{cvd}19}-1\right]E. \end{array}$$

Hence, *∂L*/*∂t* ≤ 0 if *R*_cvd19_ ≤ 1, and *∂L*/*∂t* = 0 if *E* = 0. By LaSalle's Invariance Principle, we can conclude that the DFEP of model (1) is globally asymptotically stable in *Ω*_Cvd19_ whenever *R*_cvd19_ ≤ 1.

### 4.2. Global Stability Analysis of EEP

The global asymptotic stability of *χ*_eep_^∗^ is discussed using the Lyapunov asymptotic stability theorem. From model (1), we will construct a Lyapunov function by following the study of Xu et al. [38].

**Theorem 3 .**

If *R*_cvd19_ > 1, then the endemic equilibrium point *χ*_eep_^∗^ of model (1) is globally asymptotically stable in the region *Ω*_Cvd19_.

**Proof**

First, we define*L* : {(*S*, *E*, *I*_*s*_, *I*_*a*_, *Q*, *R*, *D*) ∈ *Ω*_Cvd19_ : *S*, *E*, *I*_*s*_, *I*_*a*_, *Q*, *R*, *D* > 0} → *ℜ*.

Consider the function below:

(24) $$\begin{array}{c} L\left(S,E,I_{s},I_{a},Q,R,D\right)=\ln\left[\left(S-S_{\text{eep}}^{*}\right)+\left(E-E_{\text{eep}}^{*}\right)+\left(I_{s}-I_{s\text{eep}}^{*}\right)+\left(I_{a}-I_{a\text{eep}}^{*}\right)+\left(Q-Q_{\text{eep}}^{*}\right)+\left(R-R_{\text{eep}}^{*}\right)+\left(D-D_{\text{eep}}^{*}\right)+1\right]. \end{array}$$

This implies that *L* is *C*^1^ in the interior of *Ω*_Cvd19_, where *χ*_eep_^∗^ means the global minimum of *L* on *Ω*_Cvd19_ and *L*(*S*_eep_^∗^, *E*_eep_^∗^, *I*_*s*_^∗^_eep_, *I*_*a*_^∗^_eep_, *Q*_eep_^∗^, *R*_eep_^∗^, *D*_eep_^∗^) = 0.

The derivative of *L* along the solutions of the model in (1) is given by the expression below:

(25) $$\begin{array}{c} \dot{L}=\frac{\partial L}{\partial t}\frac{dS}{dt}+\frac{\partial L}{\partial t}\frac{dE}{dt}+\frac{\partial L}{\partial t}\frac{{dI}_{S}}{dt}+\frac{\partial L}{\partial t}\frac{{dI}_{a}}{dt}+\frac{\partial L}{\partial t}\frac{dQ}{dt}+\frac{\partial L}{\partial t}\frac{dR}{dt}+\frac{\partial L}{\partial t}\frac{dD}{dt}=\frac{\left(dS/dt\right)+\left(dE/dt\right)+\left({dI}_{S}/dt\right)+\left({dI}_{a}/dt\right)+\left(dQ/dt\right)+\left(dR/dt\right)+\left(dD/dt\right)}{\left(\left(S-S_{eep}^{*}\right)+\left(E-E_{eep}^{*}\right)+\left(I_{s}-I_{seep}^{*}\right)+\left(I_{a}-I_{aeep}^{*}\right)+\left(Q-Q_{eep}^{*}\right)+\left(R-R_{eep}^{*}\right)+\left(D-D_{eep}^{*}\right)+1\right)}. \end{array}$$

From (2), all the solutions of (11) satisfy the equality

(26) $$\begin{array}{c} N_{\text{eep}}^{*}=S_{\text{eep}}^{*}+E_{\text{eep}}^{*}+I_{s\text{eep}}^{*}+I_{a\text{eep}}^{*}+Q_{\text{eep}}^{*}+R_{\text{eep}}^{*}+D_{\text{eep}}^{*}=\frac{\rho }{\mu }. \end{array}$$

Also, *N* = *e*^−*ut*+*C*^ + *ρ*/*μ*, where *C* is the value that satisfies the condition *N*_0_ = *ρ*/*μ*.

Thus, *L* = ln(*N* − *N*^∗^ + 1) ≥ 0. Therefore,

(27) $$\begin{array}{c} \dot{L}=\frac{1}{N-\left(\rho /\mu \right)+1}\frac{dN}{dt}=\frac{\mu }{N-\left(\rho /\mu \right)+1}\left(\frac{\rho }{\mu }-N\right)\leq 0. \end{array}$$

*L* = 0 and $\dot{L}=0$ are satisfied if and only if *N* = *ρ*/*μ*.

Hence, the function $\dot{L}$ is a Lyapunov function for model (1), and the endemic equilibrium *χ*_eep_^∗^ is globally asymptotically stable by the Lyapunov asymptotic stability theorem.

## 5. Numerical Simulation

To support the mathematical analysis of model (1), the numerical simulations are carried out using the *deSolve* package [39] with the fourth-order Runge-Kutta method in RStudio programming software version 1.1.442. The simulations are divided into three parts. Part 1 is to illustrate the numerical interpretation of the disease-free and endemic equilibrium points. Part 2 is to explore the varying effects of face masks. Part 3 is to find out model (1) fitting with real data.

### 5.1. Part 1: Illustrating the Numerical Interpretation of the DFEP and EEP

The following initial conditions were used in the numerical simulations:

(28) $$\begin{array}{c} S\left(0\right)=2,150,\\ E\left(0\right)=1,750,\\ I_{S}\left(0\right)=3,930,\\ I_{a}\left(0\right)=1,965,\\ Q\left(0\right)=94,\\ R\left(0\right)=3,766. \end{array}$$

The parameter values used for the numerical simulations in Part 1 are provided in Table 3.

The results obtained from the numerical simulations are presented in Figures 2 and 3, respectively.

Figure 2 depicts a rise in the number of the susceptible population in the absence of the COVID-19 pandemic. We also note that when there is a rise in the susceptible population, the exposed population also increases. However, the increase in the exposed population is lesser compared to the susceptible population. Furthermore, no changes occurred in the quarantined and recovered population. This can be because in the absence of the COVID-19 pandemic (i.e., *I*_*s*_ = 0 and *I*_*a*_ = 0), there will be no infected population to spread the disease to the other compartments.

Figure 3 shows a slight rise in the number of individuals in the exposed compartment and a gradual reduction in the number of the infected population when necessary interventions are used as a preventive measure to reduce the spread of the COVID-19 pandemic. Additionally, there is a rise in the number of quarantined and recovered individuals from the COVID-19 pandemic. The figure also finds that if the interventions are strictly followed, it can reduce the pandemic's spread.

### 5.2. Part 2: The Varying Effects in the Use of Face Mask

The numerical simulation in Part 2 examines how varying *ψ* value affects the basic reproduction number computed in this study. As earlier defined in Table 2, *ψ* denotes the proportion of individuals who use face masks. The parameter values used in the numerical simulations for Part 2 are provided in Table 3. However, different *ψ* values (*ψ* = 0.1, 0.5, and 0.7) are considered. By computing the basic reproduction numbers and using the parameter values in Table 3, the obtained results are presented in Table 4.

From the results obtained in Table 4, it is evident that if a larger number of people consistently use face masks in a community, then the COVID-19 pandemic can be reduced.

### 5.3. Part 3: Model Fit

In this section, the real data provided in Table 5 is fitted with model (1).

The data were grouped monthly and obtained from the Department of Disease Control, Thailand [47]. The data span from January 2020 to December 2020. The monthly recorded data in Table 5 [47] were first interpolated into daily data to easily fit the real data with the simulated data. Afterward, model (1) was fitted to the daily interpolated data using a step size of 0.01. The result of the model fit is presented in Figure 4.

From Figure 4, it can be seen that the real data have two peaks which occurred on days 360 and 1,073. The model proposed in this study was able to generate the peaks obtained in the real data.

## 6. Conclusion

In this study, the nonlinear mathematical model was proposed and analyzed to understand the dynamics of the COVID-19 pandemic in Thailand. The equilibrium point relating to the formulated model was computed. Using the next generation matrix approach, the basic reproduction number denoted as relating to the model was also computed. Moreover, this study also showed that if the BRN is denoted as *R*_cvd19_ < 1, then the pandemic will die out. However, if *R*_cvd19_ > 1, then the pandemic will remain in the population.

Additionally, the global asymptotical stability of the disease-free and endemic equilibrium points has been proved. Numerical simulations were carried out to support the model analysis. The real data were also fitted to the model for predicting the infected population cases in real life. The varying effects of the use of face masks were also explored in this study, and it was found that the continuous and appropriate use of face masks can prevent the spread of the COVID-19 pandemic. Presently, the research on a vaccine to prevent the COVID-19 pandemic has yielded excellent results, with Pfizer announcing that their vaccine has a 95% efficacy. However, it will take a while before the vaccines are made readily available in all countries worldwide. Therefore, the use of face masks should be made compulsory till the vaccines are available for everyone. We propose that future researchers implement the model proposed in this study to the second wave of infected cases in Thailand to explore the efficiency of the current measures used to prevent COVID-19.

## Figures and Tables

**Figure 1:** Flowchart of the formulated model.

**Figure 2:** Simulation results of the DFEP for model (1) at different initial conditions and parameter values in Table 3 when *R*_cvd19_ = 0.28738 < 1.

**Figure 3:** Simulation results of the EEP for model (1) at different initial conditions and parameter values in Table 3 when *R*_cvd19_ = 1.40995 > 1.

**Figure 4:** The result of the model fit.

**Table 1:** Variables and their meaning used in the model.

Variables in the model	Meaning
*S*	The susceptible compartment
*E*	The exposed compartment
*I*_*s*_	The symptomatic infectious compartment
*I*_*a*_	The asymptomatic infectious compartment
*Q*	The quarantined compartment
*R*	The recovered compartment
*D*	The death compartment

**Table 2:** Parameters used in the model and their meaning.

Model parameters	Description
*ρ*	The recruitment rate into the susceptible compartment
*β*_*s*_	The effective contact rate
*β*_*a*_	The effectiveness of social distancing
*ψ*	The proportion of individuals who use a face mask
*ξ*	The efficacy of face masks
1 − *θ*	The fraction of exposed individuals who show clinical symptoms after the incubation period
*φ*	The rate of progression from the exposed compartment to the infectious compartment
*α*_*s*_	The isolation rate for individuals in the symptomatically infected compartment
*λ*_*s*_	The recovery rate of individuals in the symptomatically infected compartment
*δ*_*s*_	The COVID-19 disease mortality rate for individuals in the infectious compartment
*α*_*a*_	The isolation rate of asymptomatically infectious individuals
*λ*_*a*_	The recovery rate of asymptomatically infectious individuals
*λ*_*q*_	The recovery rate of individuals in the quarantined compartment
*δ*_*q*_	The COVID-19 disease mortality rate for individuals in the quarantined compartment
*μ*	The natural death rate of all individuals

**Table 3:** Parameter values for the numerical simulations of the DFEP and EEP.

Parameters	Parameter values for DFEP	Parameter values for EEP	Source
*ρ*	5	5	—
*β*_*s*_	Assumed	Assumed	—
*β*_*a*_	Assumed	Assumed	—
*ψ*	0.1	0.1	[40]
*ξ*	0.5	0.5	[40]
*θ*	0.5	0.5	[41–44]
*φ*	1/6	1/6	[1]
*α*_*s*_	0.2	0.2	[45]
*λ*_*s*_	1/10	1/10	[45, 46]
*δ*_*s*_	0.015	0.015	[41]
*α*_*a*_	0.2	0.2	[45]
*λ*_*a*_	1/10	1/10	[45, 46]
*λ*_*q*_	0.05	0.05	[45, 46]
*δ*_*q*_	0.015	0.015	[41]
*μ*	3.6529 × 10^−5^	3.6529 × 10^−5^	[47]
Basic reproduction number	*R*_cvd19_ = 0.28738 < 1	*R*_cvd19_ = 1.40995 > 1	

**Table 4:** Numerical simulation of the varying effects of the parameter *ψ*.

Parameters	Parameter value	*R*_cvd19_
*ψ*	0.1 (10%)	1.40995 > 1
*ψ*	0.5 (50%)	0.62111 < 1
*ψ*	0.7 (70%)	0.00332 < 1

**Table 5:** Number of recorded COVID-19 cases in Bangkok, Thailand, from January 2020 to December 2020.

Month	Number of infected population recorded
January 2020	19
February 2020	23
March 2020	1609
April 2020	1303
May 2020	127
June 2020	90
July 2020	139
August 2020	102
September 2020	152
October 2020	216
November 2020	218
December 2020	1509

## Data Availability

The data used to support the findings of this study are included within the article.
